# Advanced Glycation End-Products Enhance Lung Cancer Cell Invasion and Migration

This article has been retracted.

**DOI:** 10.3390/ijms17081289

**Published:** 2016-08-09

**Authors:** Te-Chun Hsia, Mei-Chin Yin, Mei-Chin Mong

**Affiliations:** 1 Department of Respiratory Therapy, China Medical University, 40402 Taichung City, Taiwan; derrick.hsia@msa.hinet.net; 2 Department of Internal Medicine, China Medical University Hospital, 40402 Taichung City, Taiwan; 3 Department of Nutrition, China Medical University, 40402 Taichung City, Taiwan; 4 Department of Health and Nutrition Biotechnology, Asia University, 41354 Taichung City, Taiwan; mmong@asia.edu.tw

**Keywords:** CML, pentosidine, non-small cell lung cancer, migration, invasion

## Abstract

Effects of carboxymethyllysine (CML) and pentosidine, two advanced glycation end-products (AGEs), upon invasion and migration in A549 and Calu-6 cells, two non-small cell lung cancer (NSCLC) cell lines were examined. CML or pentosidine at 1, 2, 4, 8 or 16 μmol/L were added into cells. Proliferation, invasion and migration were measured. CML or pentosidine at 4–16 μmol/L promoted invasion and migration in both cell lines, and increased the production of reactive oxygen species, tumor necrosis factor-α, interleukin-6 and transforming growth factor-β1. CML or pentosidine at 2–16 μmol/L up-regulated the protein expression of AGE receptor, p47^phox^, intercellular adhesion molecule-1 and fibronectin in test NSCLC cells. Matrix metalloproteinase-2 protein expression in A549 and Calu-6 cells was increased by CML or pentosidine at 4–16 μmol/L. These two AGEs at 2–16 μmol/L enhanced nuclear factor κ-B (NF-κ B) p65 protein expression and p38 phosphorylation in A549 cells. However, CML or pentosidine at 4–16 μmol/L up-regulated NF-κB p65 and p-p38 protein expression in Calu-6 cells. These findings suggest that CML and pentosidine, by promoting the invasion, migration and production of associated factors, benefit NSCLC metastasis.

## 1. Introduction

Advanced glycation end-products (AGEs) such as carboxymethyllysine (CML) and pentosidine are reactive compounds formed from glycosylation of sugars and macromolecules like proteins or lipids. CML and pentosidine could be endogenously synthesized under certain pathological conditions such as diabetes or Alzheimer’s disease, and these AGEs are considered as endogenous AGEs. Many foods including sauces, canned meats, nuts or grain products contain CML, pentosidine and other AGEs [1,2]. Thus, these foods are an exogenous source of AGEs. It is reported that dietary intake of AGEs-rich foods increased circulating AGE levels in patients with diabetes or chronic kidney disease [3,4]. So far, the impact of endogenous or exogenous AGEs upon cancer progression has been a focus because AGE levels were found to be markedly elevated in both serum and tumors, especially in more aggressive tumors [5]. Kim et al. [6] and Sharaf et al. [7] indicated that the engagement of AGEs with their receptor (RAGE) further up-regulated RAGE protein expression, and subsequently activated mitogen-activated protein kinase (MAPK) and nuclear factor-κB (NF-κB) signaling pathways in myeloid leukemia and breast cancer cells.

The studies of Weng et al. [8] and Tsao et al. [9] revealed that the activation of MAPK and NF-κB pathways in non-small cell lung cancer (NSCLC) cells promoted the massive production of oxidative, inflammatory and angiogenic factors including reactive oxygen species (ROS), tumor necrosis factor (TNF)-α, intercellular adhesion molecule (ICAM)-1, transforming growth factor (TGF)-β1, vascular endothelial growth factor (VEGF), fibronectin and matrix metalloproteinases (MMPs). Moreover, higher TGF-β1, ICAM-1 and MMP-2 levels in circulation and/or lung tissue were correlated with poor prognosis in NSCLC patients [10,11]. Actually, RAGE is constitutively expressed in lung tissue [12]. However, Marinakis et al. [13] reported that RAGE expression was lower in tumor of NSCLC, the most common type of lung cancer. Those authors indicated that the reduction of RAGE expression might contribute to interrupt cell-to-cell or cell-to-substrate communication, which favored cancer cell progression and migration. Therefore, it is highly possible that the presence of exogenous and/or endogenous AGEs, through rapidly stimulating RAGE expression and activating associated signaling pathways, may enhance the generation of oxidative, metastatic and inflammatory factors, and promote NSCLC progression. Takino et al. [14] indicated that RAGE was associated with cancer malignancy, and glyceraldehyde-derived AGEs facilitated the migration and invasion of A549 cells by activating Rac 1 and increasing ROS formation. Obviously, the influence of AGEs upon NSCLC progression could not be ignored. Since CML and pentosidine are two common AGEs in foods [1], the effects and action modes of these two AGEs upon NSCLC development are worthy of investigation. If CML and/or pentosidine benefit the proliferation, invasion and/or migration of NSCLC cells, they benefit NSCLC progression and deterioration.

A549 and Calu-6 cells are human NSCLC cell lines, and have been widely used for NSCLC cell model researches [9,14]. In our present study, these two cell lines were also used to examine the effects of CML and pentosidine at various concentrations upon NSCLC cell proliferation, invasion and migration. Furthermore, the impact of these AGEs upon protein expression of RAGE, TGF-β1, ICAM-1, MMP-2, NADPH oxidase, NF-κB and MAPK was evaluated in order to understand the possible modes of action of AGEs upon NSCLC.

## 2. Results

### 2.1. Effects of CML and Pentosidine upon Invasion and Migration of Lung Cancer Cells

As shown in Table 1 and Figure 1, CML or pentosidine treatments at test concentrations did not affect proliferation, and protein expression of Bcl-2, Bax, caspase-3 or caspase-8 in A549 cells and Calu-6 cells (*p* > 0.05). However, CML or pentosidine at 4–16 μmol/L enhanced invasion and migration of A549 cells (Table 2, *p* < 0.05). In Calu-6 cells, these two AGEs at 2–16 μmol/L promoted invasion and migration (*p* < 0.05).

### 2.2. Effects of CML and Pentosidine upon Oxidative and Inflammatory Factors

CML at 4–16 μmol/L and pentosidine at 2–16 μmol/L increased the production of ROS, TNF-α, IL-6 and TGF-β1 in A549 and Calu-6 cells (Table 3, *p* < 0.05). Concentration-dependent manner was presented in raising TNF-α and TGF-β1 release in test cells (*p* < 0.05). CML at 4–16 μmol/L and pentosidine at 2–16 μmol/L up-regulated RAGE expression in A549 and Calu-6 cells (Figure 2, *p* < 0.05). In both cell lines, p47^phox^ protein expression was enhanced by CML or pentosidine at 2–16 μmol/L (*p* < 0.05). However, CML or pentosidine at test concentrations did not alter gp91^phox^ protein expression in two NSCLC cell lines (*p* > 0.05).

### 2.3. Effects of CML and Pentosidine upon VEGF, ICAM-1, Fibronectin, MMP-2 and MMP-9 Expression

As shown in Figure 3, CML or pentosidine at 2–16 μmol/L up-regulated ICAM-1 and fibronectin protein expression in A549 and Calu-6 cells (*p* < 0.05). MMP-2 protein expression in A549 cells was increased by two AGEs at 4–16 μmol/L (*p* < 0.05). In Calu-6 cells, CML or pentosidine at 2–16 μmol/L enhanced MMP-2 protein expression (*p* < 0.05). CML and pentosidine at test concentrations did not change VEGF and MMP-9 protein expression in test NSCLC cell lines (*p* > 0.05).

### 2.4. Effects of CML and Pentosidine upon NF-κB and MAPK Pathways

In A549 cells, CML or pentosidine at 2–16 μmol/L up-regulated NF-κB p65 protein expression (Figure 4, *p* < 0.05). These two AGEs at 1–16 μmol/L increased p38 phosphorylation in A549 cells (*p* < 0.05). In Calu-6 cells, CML and pentosidine promoted NF-κB p65 protein expression at 2–16 μmol/L and 4–16 μmol/L, respectively (*p* < 0.05). CML and pentosidine at 2–16 μmol/L enhanced p-p38 protein expression in Calu-6 cells (*p* < 0.05). CML and pentosidine at test concentrations failed to affect NF-κB p50, JNK and ERK1/2 protein expression or phosphorylation in test NSCLC cell lines (*p* > 0.05). As shown in Figure 5, CML and pentosidine at 2–16 μmol/L increased NF-κB p50/65 DNA binding activity in A549 and Calu-6 cells (*p* < 0.05).

## 3. Discussion

Many foods, especially high temperature treated foods, have substantial levels of CML, pentosidine or other AGEs [15,16]. Furthermore, CML and/or pentosidine levels in human circulation could be increased by dietary intake of AGE-containing foods [3,4]. Consequently, these AGEs present in circulation could interact with cancer cells in lung tissue. Turner et al. [5] indicated that exogenous AGEs were linked to cancer risk and disparity. In our present study, CML and pentosidine at test concentrations did not alter cell proliferation and protein expression of Bcl-2, Bax, caspase-3 and caspase-8, apoptotic biomarkers, in two NSCLC cell lines. It seems that these AGEs at those concentrations might not be able to stimulate or inhibit lung tumor growth. However, we found that CML or pentosidine promoted invasion and migration, increased ROS and inflammatory cytokines production, up-regulated protein expression of RAGE, p47^phox^, ICAM-1, fibronectin and MMP-2, as well as activated NF-κB and MAPK pathways in A549 and Calu-6 cells. These findings suggest that these two AGEs might benefit NSCLC metastasis. Sharaf et al. [7] and Ko et al. [17] reported that AGEs enhanced proliferation, invasion and migration in oral and breast cancer cells. The study of Takino et al. [14] revealed that glyceraldehyde-derived AGEs at 20–100 μg/mL increased the migration capacity of A549 cells. Thus, our findings agreed and suggested that CML and pentosidine are promotive agents upon lung cancer cell migration and invasion.

NADPH oxidase complex is responsible for ROS generation in lung tissue. Excessive ROS formation due to NADPH oxidase activation facilitates lung tumorigenesis [18,19]. Our data revealed that CML and pentosidine markedly up-regulated protein expression of p47^phox^, a cytosolic component of NADPH oxidase, in test NSCLC cells, which subsequently increased ROS production. TGF-β1 is an inflammatory mediator, and also an angiogenic inducer because it enhances epithelial-to-mesenchymal transition in late-stage tumor progression [20]. Saji et al. [21] indicated that TGF-β1, via its immunosuppressive action, facilitated pulmonary metastasis in NSCLC patients. Thus, the greater ROS and TGF-β1 production in CML or pentosidine treated A549 or Calu-6 cells partially explained that these AGEs enhanced oxidative, inflammatory and angiogenic stress in those cells, which might in turn favor the development of microvascular permeability and metastatic actions in lung cancer.

Our Western blot data indicated that CML and pentosidine upregulated protein expression of RAGE, MAPK and NF-κB in two NSCLC cell lines. It is reported that the interaction between RAGE and AGEs could activate MAPK and NF-κB signaling pathways [22]. However, we found that CML or pentosidine at 1 μmol/L increased p38 phosphorylation in A549 cells, and both AGEs at 2 μmol/L up-regulated NF-κB p65 expression in A549 and Calu-6 cells; but CML at 4 μmol/L raised RAGE expression in two NSCLC cell lines. These findings suggest that these AGEs might be able to directly mediate NF-κB and MAPK expression, not RAGE dependent. In addition, CML or pentosidine treatments also elevated NF-κB p50/65 DNA binding activity in A549 and Calu-6 cells, which supported the activation of NF-κB. It is known that the activation of these pathways promotes the transcription of their target molecules including oxidants, inflammatory cytokines and even metastatic factors, and finally contributes to lung cancer migration and invasion [23]. Since CML and pentosidine markedly activated RAGE, NF-κB and MAPK pathways in test NSCLC cells, it was reasonable to observe the over-production of ROS, TGF-β1, TNF-α and IL-6 in those NSCLC cells. Besides MAPK and NF-κB pathways, Bao et al. [24] reported that AGE–RAGE interaction promoted prostate cancer cell proliferation via activating PI3K/Akt signaling pathway. Thus, it is highly possible that other pathways are involved in AGEs’ induced NSCLC progression. On the other hand, RAGE could bind to other ligands like HMGB1 and S100P, which subsequently activated TLR-4 and PI3K-Akt pathways, and favored lung cancer progression [25,26]. Thus, the up-regulated RAGE due to CML or pentosidine might in turn benefit NSCLC deterioration through engaging with other ligands and accelerating oxidative, inflammatory, angiogenic and metastatic reactions. Therefore, lowering exogenous AGEs via dietary restriction might be able to reduce RAGE protein expression, diminish the interaction of AGEs and RAGE, and decrease the formation of contributors toward NSCLC metastasis.

ICAM-1, a cell adhesion factor, participates in intercellular and cell-extracellular matrix interactions of cancer cells [27]. It is reported that NSCLC patients had higher circulating ICAM-1 levels [28,29], which reflected poor prognosis and worse survival in those patients [28]. Fibronectin is an extra cellular matrix glycoprotein. The expression of fibronectin is increased with lung tumor growth, and is highly associated with resistance to lung cancer therapy [30]. MMPs degrade extracellular matrix components and allow cancer cells to approach vascular and lymphatic systems [31]. MMP-2 could demote type IV collagen, the basic component of the basement membrane in extracellular matrix [32]. We found that CML or pentosidine treatments markedly increased ICAM-1, fibronectin and MMP-2 protein expression in two NSCLC cell lines. Since those metastatic factors had been up-regulated, the observed greater invasion and migration in those cells could be explained. In addition, we notified that CML or pentosidine at test concentrations failed to affect VEGF and MMP-9, two crucial factors responsible for cancer metastasis. These results implied that those AGEs selectively mediated some molecules to promote the invasion and migration in those NSCLC cells.

It is interesting to find that pentosidine at 4–16 μmol/L caused greater generation of ROS, TNF-α, IL-6 and TGF-β1 than CML at equal concentrations in A549 and Calu-6 cells. Also, pentosidine at 8 and 16 μmol/L induced greater RGAE protein expression than CML in those NSCLC cells. It is likely that pentosidine was more reactive than CML toward NSCLC cells. Consequently, pentosidine at 8 or 16 μmol/L led to greater migration than CML in A549 and Calu-6 cells. Although CML and pentosidine are AGEs, their impact upon those NSCLC cells does not seem to be identical.

## 4. Materials and Methods

### 4.1. Materials

CML (95%) and pentosidine (90%) were purchased from Cayman Chemical Co. (Ann Arbor, MI, USA). Plates, medium, chemicals and antibiotics used for cell culture were purchased from Difco Laboratory (Detroit, MI, USA). Human lung cancer cell lines, A549 and Calu-6, were obtained from American Type Culture Collection (Rockville, MD, USA).

### 4.2. Cell Culture

Cells were cultured in RPMI 1640 medium, containing 10% fetal bovine serum (FBS), 100 units/mL of penicillin and 100 units/mL of streptomycin (pH 7.4) at 37 °C in 5% CO_2_. The culture medium was changed every three days, and cells were subcultured once a week. A phosphate buffer saline (PBS, pH 7.2) was added to adjust the cell number to 10^5^/mL for various experiments and analyses. The plasma concentrations of CML and pentosidine in healthy people were in the range of 0.053–0.49 μmol/L [33]. However, plasma level of these two AGEs in patients with diabetes or renal failure was in the range of 0.2–12.6 μmol/L [34,35]. Thus, CML or pentosidine at 1, 2, 4, 8 and 16 μmol/L were used in present study in order to examine the adverse and possible pathological impact of AGEs. Cells were treated with CML or pentosidine at those concentrations for 18 h at 37 °C, which resulted in 96.3% ± 2.1% incorporation of test agents. AGEs treated cells were washed twice by PBS. CML or pentosidine concentration in collected PBS was analyzed by a competitive ELISA kit (Roche Diagnostics, Penzberg, Germany) or HPLC method of Miyata et al. [35]. The left AGEs in cells were defined as incorporated. Our preliminary test showed that 6, 12, 18, 24 or 36 h incubation led to 43.2%, 68.4%, 96.5%, 95.4% and 94.2% incorporation of CML or pentosidine. Thus, 18 h incubation was used for this study. Control group contained no CML or pentosidine.

### 4.3. Cell Proliferation

Cell proliferation was determined by using a bromodeoxyuridine ELISA colorimetric assay (Roche Diagnostics, Indianapolis, IN, USA). Cells were counted by using a hemocytometer.

### 4.4. Cell Invasion and Migration

Cell invasion and migration were measured in transwell chambers by matrigel- and fibronectin-coated polycarbonate filters, respectively. In brief, cells (10^5^/100 μL) were seeded into the upper chamber in 200 μL of serum-free medium; and the lower chamber was filled with 0.66 mL of RPMI 1640 media containing 10% of FBS as a chemoattractant. After 6 h incubation for migration assay or 16 h incubation for invasion assay at 37 °C, the cells on the upper surface of the filter were removed by a cotton swab. The migrated or invaded cells to the lower surface of the filter were stained with 0.2% crystal violet in 10% ethanol. Four independent fields of invasive or migratory cells per well were photographed under the microscope to count the cell numbers. Data were calculated as a percentage of the control groups.

### 4.5. Measurement of ROS, Interleukin (IL)-6, TNF-α and TGF-β1

Cells were washed and suspended in RPMI 1640 medium. ROS level was determined by 2’,7’-dichlorofluorescein diacetate, an oxidation sensitive dye. Cells were incubated with 50 μmol/L dye for 30 min and washed twice with PBS. After centrifugation at 412× *g* for 10 min, the medium was removed and cells were dissolved by 1% Triton X-100. Fluorescence value was measured at time 0 and 5 min by using a fluorescence microplate reader at excitation and emission wavelengths at 485 and 530 nm, respectively. Relative fluorescence unit (RFU) was the difference in fluorescence values obtained between time 0 and 5 min. Results are expressed as RFU/mg protein. The levels of IL-6, TNF-α and TGF-β1 in cell culture supernatant were measured by ELISA kits (R&D Systems, Minneapolis, MN, USA). Protein concentration was determined by an assay kit (Pierce Biotechnology Inc., Rockford, IL, USA), and bovine serum albumin was used as a standard.

### 4.6. Assay for NF-κB p50/65 DNA Binding Activity

Nuclei pellets were isolated and re-suspended in a solution containing 20 mM HEPES, 1 mM EDTA, 0.4 M NaCl, 1 mM DTT and 25% glycerol. After incubation and centrifugation, supernatants were collected for protein concentration quantification by protein assay reagents (Bio-Rad Laboratories Inc., Hercules, CA, USA). NF-κB p50/65 DNA binding activity was determined by an assay kit (Chemicon International Co., Temecula, CA, USA). The binding of activated NF-κB was processed by a primary polyclonal antibody against NF-κB p50/p65, and followed by treating with an antibody conjugated with horseradish peroxidase. 3,3′,5,5′-tetramethylbenzidine was the substrate. The absorbance at 450 nm was recorded. Data are shown as optical density (OD)/mg protein.

### 4.7. Western Blot Analyses

Cell was homogenized in protease-inhibitor cocktail containing 0.5% Triton X-100 (Sigma-Aldrich Chemical Co., St. Louis, MO, USA). This homogenate was further mixed with a buffer composed of 60 mM Tris-HCl, 2% β-mercaptoethanol and 2% SDS (pH 7.2), and boiled for 5 min. Sample at 40 μg protein was applied to 10% SDS-PAGE, and further transferred to a nitrocellulose membrane (Millipore, Bedford, MA, USA) for 1 h. After blocking with a solution containing 5% skim milk for 1 h to prevent non-specific binding of antibody, membrane was reacted with monoclonal antibody against Bcl-2, Bax, caspase-3, caspase-8 (1:1000), RAGE (1:500), p47^phox^, gp91^phox^, VEGF, ICAM-1, MMP-2, MMP-9, fibronectin, NF-κB (1:1000) or MAPK (1:2000) (Boehringer-Mannheim, Indianapolis, IN, USA) at 4 °C overnight, and followed by treating samples with horseradish peroxidase-conjugated antibody for 3.5 h at room temperature. Glyceraldehyde-3-phosphate dehydrogenase (GAPDH) was used as a loading control, and the detected bands were quantified by normalizing against GAPDH.

### 4.8. Statistical Analysis

The effect of each treatment was analyzed from 10 different preparations (*n* = 10). Data were expressed as means ± standard deviation (SD), and processed for analysis of variance. Differences among means were determined by Fisher’s Least Significance Difference Test with significance defined at *p* < 0.05.

## 5. Conclusions

CML and pentosidine enhanced invasion and migration of A549 and Calu-6 cells. These AGEs increased the production of ROS and inflammatory cytokines, and up-regulated protein expression of NADPH oxidase, RAGE, ICAM-1, fibronectin, MMP-2, NF-κB p65 and p-p38 in both NSCLC cell lines. These findings suggest that CML and pentosidine benefit NSCLC metastasis.

## Figures and Tables

**Figure 1:** Effects of CML or pentosidine at 0 (control), 1, 2, 4, 8 or 16 μmol/L upon protein expression of Bcl-2, Bax, caspase-3 and caspase-8 in human A549 and Calu-6 cells. Cells were exposed to CML or pentosidine for 18 h at 37 °C. Data are mean ± SD (*n* = 10).

**Figure 2:** Effects of CML or pentosidine at 0 (control), 1, 2, 4, 8 or 16 μmol/L upon protein expression of RAGE, p47^phox^ and gp91^phox^ in human A549 and Calu-6 cells. Cells were exposed to CML or pentosidine for 18 h at 37 °C. Data are mean ± SD (*n* = 10) and shown in the following table. ^a–d^ Means within a column without a common letter differ, *p* < 0.05.

**Figure 3:** Effects of CML or pentosidine at 0 (control), 1, 2, 4, 8 or 16 μmol/L upon protein expression of VEGF, ICAM-1, fibronectin, MMP-2 and MMP-9 in human A549 and Calu-6 cells. Cells were exposed to CML or pentosidine for 18 h at 37 °C. Data are mean ± SD (*n* = 10) and shown in the following table. ^a–e^ Means within a column without a common letter differ, *p* < 0.05.

**Figure 4:** Effects of CML or pentosidine at 0 (control), 1, 2, 4, 8 or 16 μmol/L upon protein expression of NF-κB and MAPK in human A549 and Calu-6 cells. Cells were exposed to CML or pentosidine for 18 h at 37 °C. Data are mean ± SD (*n* = 10), and shown in the following table. ^a–e^ Means within a column without a common letter differ, *p* < 0.05.

**Figure 5:** Effects of CML or pentosidine at 0 (control), 1, 2, 4, 8 or 16 μmol/L upon NF-κB p50/65 DNA binding activity, determined as OD450 nm/mg protein, in human A549 and Calu-6 cells. Cells were exposed to CML or pentosidine for 18 h at 37 °C. Data are mean ± SD (*n* = 10). ^a–e^ Means among bars without a common letter differ, *p* < 0.05.

**Table 1:** Effects of CML or pentosidine at 0 (control), 1, 2, 4, 8 or 16 μmol/L upon cell proliferation (% of control) in human A549 and Calu-6 cells. Cells were exposed to CML or pentosidine for 18 h at 37 °C. Data are mean ± SD (*n* = 10).

	A549 Cells	Calu-6 Cells
CML, 0	100	100
1	98 ± 4	101 ± 2
2	101 ± 5	97 ± 4
4	103 ± 3	100 ± 3
8	97 ± 5	103 ± 2
16	102 ± 4	99 ± 4
Pentosidine, 0	100	100
1	102 ± 3	99 ± 5
2	103 ± 4	102 ± 2
4	100 ± 2	104 ± 3
8	97 ± 3	101 ± 4
16	101 ± 5	98 ± 5

**Table 2:** Effects of CML or pentosidine at 0 (control), 1, 2, 4, 8 or 16 μmol/L upon cell invasion (% of control) and migration (% of control) in human A549 and Calu-6 cells. Cells were exposed to CML or pentosidine for 18 h at 37 °C. Data are mean ± SD (*n* = 10). ^a–e^ Means within a column without a common letter differ, *p* < 0.05.

	A549 Cells		Calu-6 Cells	
	Invasion	Migration	Invasion	Migration
CML, 0	100 ^a^	100 ^a^	100 ^a^	100 ^a^
1	102 ± 3 ^a^	98 ± 4 ^a^	99 ± 2 ^a^	98 ± 5 ^a^
2	107 ± 4 ^a^	106 ± 5 ^a^	127 ± 4 ^b^	132 ± 3 ^b^
4	135 ± 3 ^b^	140 ± 7 ^b^	155 ± 5 ^c^	158 ± 4 ^c^
8	142 ± 5 ^b^	144 ± 5 ^b^	182 ± 4 ^d^	187 ± 6 ^d^
16	166 ± 7 ^c^	174 ± 4 ^c^	190 ± 6 ^d^	195 ± 5 ^d^
Pentosidine, 0	100 ^a^	100 ^a^	100 ^a^	100 ^a^
1	99 ± 2 ^a^	104 ± 5 ^a^	103 ± 4 ^a^	107 ± 4 ^a^
2	103 ± 5 ^a^	108 ± 3 ^a^	133 ± 2 ^b^	147 ± 3 ^b^
4	138 ± 4 ^b^	142 ± 4 ^b^	164 ± 5 ^c^	173 ± 6 ^c^
8	157 ± 5 ^c^	168 ± 6 ^c^	191 ± 7 ^d^	205 ± 5 ^d^
16	184 ± 7 ^d^	201 ± 4 ^d^	225 ± 6 ^e^	232 ± 3 ^e^

**Table 3:** Effects of CML or pentosidine at 0 (control), 1, 2, 4, 8 or 16 μmol/L upon ROS (RFU/mg protein), TNF-α (pg/mg protein), IL-6 (pg/mg protein) and TGF-β1 (pg/mg protein) levels in human A549 and Calu-6 cells. Cells were exposed to CML or pentosidine for 18 h at 37 °C. Data are mean ± SD (*n* = 10). ^a–e^ Means within a column without a common letter differ, *p* < 0.05.

	A549 Cells				Calu-6 Cells			
	ROS	TNF-α	IL-6	TGF-β1	ROS	TNF-α	IL-6	TGF-β1
CML, 0	1.97 ± 0.18 ^a^	156 ± 13 ^a^	133 ± 10 ^a^	141 ± 8 ^a^	2.09 ± 0.21 ^a^	160 ± 18 ^a^	136 ± 8 ^a^	130 ± 7 ^a^
1	2.06 ± 0.21 ^a^	161 ± 9 ^a^	142 ± 8 ^a^	147 ± 5 ^a^	2.14 ± 0.15 ^a^	158 ± 12 ^a^	142 ± 14 ^a^	139 ± 10 ^a^
2	2.18 ± 0.25 ^a^	167 ± 17 ^a^	150 ± 16 ^a^	163 ± 11 ^a^	2.23 ± 0.24 ^a^	166 ± 9 ^a^	148 ± 10 ^a^	145 ± 12 ^a^
4	2.65 ± 0.17 ^b^	194 ± 14 ^b^	187 ± 11 ^b^	197 ± 9 ^b^	2.71 ± 0.17 ^b^	201 ± 15 ^b^	191 ± 16 ^b^	186 ± 8 ^b^
8	2.84 ± 0.20 ^b^	237 ± 22 ^c^	224 ± 19 ^c^	245 ± 13 ^c^	3.18 ± 0.23 ^c^	242 ± 13 ^c^	247 ± 19 ^c^	217 ± 14 ^c^
16	3.39 ± 0.28 ^c^	280 ± 19 ^d^	275 ± 23 ^d^	291 ± 17 ^d^	3.30 ± 0.28 ^c^	293 ± 20 ^d^	258 ± 25 ^c^	266 ± 21 ^d^
Pentosidine, 0	2.08 ± 0.11 ^a^	149 ± 15 ^a^	136 ± 7 ^a^	139 ± 9 ^a^	2.21 ± 0.14 ^a^	152 ± 12 ^a^	130 ± 11 ^a^	134 ± 9 ^a^
1	2.13 ± 0.16 ^a^	157 ± 12 ^a^	145 ± 14 ^a^	148 ± 10 ^a^	2.18 ± 0.19 ^a^	159 ± 8 ^a^	127 ± 14 ^a^	143 ± 13 ^a^
2	2.62 ± 0.09 ^b^	188 ± 10 ^b^	176 ± 18 ^b^	182 ± 13 ^b^	2.57 ± 0.12 ^b^	195 ± 16 ^b^	178 ± 15 ^b^	175 ± 15 ^b^
4	2.75 ± 0.21 ^b^	226 ± 19 ^c^	213 ± 15 ^c^	234 ± 8 ^c^	3.06 ± 0.20 ^c^	240 ± 23 ^c^	201 ± 19 ^b^	223 ± 10 ^c^
8	3.55 ± 0.18 ^c^	270 ± 22 ^d^	259 ± 17 ^d^	290 ± 14 ^d^	3.59 ± 0.16 ^d^	291 ± 26 ^d^	263 ± 25 ^c^	279 ± 14 ^d^
16	3.69 ± 0.25 ^c^	331 ± 27 ^e^	304 ± 22 ^e^	359 ± 19 ^e^	3.74 ± 0.25 ^d^	355 ± 21 ^e^	310 ± 27 ^d^	348 ± 16 ^e^

## Abbreviations

CML	carboxymethyllysine
AGE	advanced glycation end-product
NSCLC	non-small cell lung cancer
MMP	matrix metalloproteinase
RAGE	receptor for advanced glycation end-product
MAPK	mitogen-activated protein kinase
NF-κB	nuclear factor κ-B
ROS	reactive oxygen species
TNF	tumor necrosis factor
ICAM	intercellular adhesion molecule
TGF	transforming growth factor
VEGF	vascular endothelial growth factor
